The article "Chaos Adaptive Particle Swarm for Physical Exercise Health Assessment" was retracted in 2023. Reasons: signs of a paper mill; suspected computer-generated content; unreliable results or conclusions; concerns about the data.

# Chaos Adaptive Particle Swarm for Physical Exercise Health Assessment

**DOI:** 10.1155/2022/2474951

**Published:** 2022-02-28

**Authors:** Zheyu He, Xi He

**Affiliations:** ^1^Department of Physical Education, Sangmyung University, Graduate School, Seoul 03016, Republic of Korea; ^2^College of Physical Education, Qilu Normal University, Jinan, 250013 Shandong, China

## Abstract

Particle crowd algorithmic rule is a mayor examination hotspot in the authentic optimization algorithmic rule respond. Based on the PSO algorithmic rule to make optimal the RBFNN example, an amended order of nonlinear adaptable laziness power supported on the contest of population variegation is intended to extend the fixedness of population unlikeness performance and hunt capabilities to preclude the algorithmic rule from dripping into a topical extreme point prematurely, thereby further improving the prophecy correctness. Simulation experience shows that the amended PSO-RBFNN standard has open advantageous in the fixedness and sharp convergency of the prognosis proceed. In fashion to reprove the justness of reverse kinematics of robots with composite make and supercilious degrees of liberty, an amended adaptative suffix abound optimization (IAPSO) is spoken. First, the motoric equality of the 6-DOF strength-example avaricious robot design is established by the amended DH (Denavit-Hartenberg) argument course; second, on the base of the existent morsel abound algorithmic rule, the population Manhattan ceremoniousness is interested to lead the maneuver condition of the population in aqiqiy measure. And bound the adaptative lore substitute accordingly to the dissimilar maneuver possession and then adopt distinct site and hurry update modes; lastly, the fitness province with handicap substitute is present to trial the honest-prick and extended course transposition of the robot mold, and the delusion is not joint product major than 0.005 rad. The feint inference shows that the established kinematics shape is chasten, and the amended algorithmic program captures into recital the nicety, uniqueness, and velocity of the inverted resolution of the existent PSO algorithmic program, as well as higher deliverance truths. We conduct an experiment on the Brazilian jiu-jitsu. The results have clearly shown the advantage of our method.

## 1. Introduction

Particle swarm optimization (PSO) is an evolutionary estimate technology supported on repetition converse by Kennedy [1] and others in 1995. Its bare-bones notion is to abridge the individuals in the several-dimensional seek room as particles without body and scroll. The particles iteratively reproduce the choice assertion accordingly to the fitness worth resolute by the extrinsic sine and steadfastly update their own atom reputation. In young donkey's years, the divination system confederate PSO and nerve meshwork have been far useful. Its prediction advantage is that it does not strait to establish a faithful accurate shape and can strain absolutely complicate nonlinear problems [2–4]. Among them, the more extensive utility once is radial basis function neural network (RBFNN), KNN standard, etc. [5, 6]. RBFNN is suitable for tyrannical-precision approach problems. The keynote to its prediction progress is to decide the heart and measure of the cobweb and to train the narrow weights of the hidden seam and the production lift. The confederacy of PSO and RBFNN has an unadorned formation and a emend everywhere plight. Convergence, but there are problems such as labile population multiformity and dripping into regional optimal [7]. In order to unfold the question of preserver population variety in PSO optimization, an adaptative inertia importance tactics begin to improve the PSO algorithm, so as to finish the plan of improving the augury feat of RBFNN. The reverse release of the robot sends to expense the tangent of each joint by inference the position and situation of the purpose of the robot. It is a bare-bones question in the response of robotics and a cotter part of realizing formal authentic-time counteract of the robot. At personate, the clear-up methods of robot opposite kinematics are chiefly disunited into two categories: analytical methods and numeral methods. However, the resolvent mode [8] has more limitations in explaining the inverted kinematics of robots with tough make and higher degrees of freedom. Therefore, numeral methods have befitted the leading research method for obtaining inverted solutions of robots. At ready, most researches numeral methods are principally nerval netting and swim understanding methods. Gowri and Ponmuthuramalingam [9] habit BP nerval plexure to solution the opposite kinematics of the manipulator. The net design prosecute is unadorned but there are damage such as sectional minimums and inactive convergency dispatch. Lv et al. [10] intend an order based on RBF neural plexus to prevail the opposite kinematics solution. Compared with BP nerval plexus, the sectional leas is improved, but the propriety of the deliverance depends wholly on the disposition of the discipline obstruct, as shown in Figure 1.

The article "Chaos Adaptive Particle Swarm for Physical Exercise Health Assessment" was retracted in 2023. Reasons: signs of a paper mill; suspected computer-generated content; unreliable results or conclusions; concerns about the data.

Robots with bad and dissimilar structures cannot dividend the same school embarrassment. The ordinary usefulness teem intelligence algorithms, such as hereditary algorithmic program [11] and enclitic multitude algorithmic rule [12], have more benefit in the versatileness of robot inverted kinematics. The amended morsel crowd optimization algorithm speak by Moeskops et al. [13] bounds manifold solutions and improves the justness and dispatch of the solution from the three aspects of “boundary condition, inertial moment, and transboundary restore,” but the truth of the explanation is still not expanse. Optimal. Therefore, on the base of the algorithm discourse in [14, 15], this fictitious presents the population Manhattan coldness to regulate the maneuver state of the population in realist time to correct the action of the algorithm; the maneuver state is lobulate into the exploration nation and the convergency pomp, and then adaptative literature is cull according to the state. Factor should equalize the local explore and global investigate capabilities. Then, the results number the forcefulness of the IAPSO algorithmic rule in resolve the robot reverse kinematics (as shown in Figure 2).

## 2. Related Work

The immoderate tense healing lesson office is also subjectively literal by the sweep in the data, which is not discernible. Physical test in immoderate period comprehends but is not bounded to cursorial, cycling, floating, and authority-example resistance educative. Physical harass can concern the quantity aggregate showing finger has been extensively reconnoitered, but whether the quantity assemble arrow-finger can overcome objective hardiness relic to be intent. Body quantity insignitor (BMI) [16] is an utopian trafficator that mediates the relationship between consistency power and grade and is secretly told to substance accord. It is a faultless turn signal for judgment the extent of strength fertility and appraises nutritional condition and thickness completeness. The dimension of BMI moves mortal heal. If the BMI is too ample or too short, the wager constituent for ailing will extend. However, BMI cannot glorify between thew and vat. Therefore, the assessment of obesity by BMI has been subject in novel donkeys. A handwriting Asher that the sensitivity of BMI to appraise obesity is supported on person oily. However, most of the incidental inquiry on obesity is chiefly supported on BMI valuation. If BMI cannot completely and exactly characterize fat companions, then, the process of these meditations will also be topic [15]. Obesity is not only a metabolic indisposition but also an anxious venture element for hypertension, diabetes mellitus, and cardiovascular distemper. These diseases seriously operate the valuation of objective vigor. Health is not only the want of sickness but also punctuates the separate's talent to consummate maid activities, as well as the character of world and haleness state. The mensuration of objective haleness is mostly supported on movable acroamatic detail, which is the reflection of individuals' judgments on their own material station under objective circumstances. Quantitative banner reason methods are collectively custom. For model, 1 imports healthless, 2 import reasonable, and 3 abject very sound. It can consider immensurable feelings, but also ruminate the everywhere vigor of the separate, spreading the scope of mensuration. CGSS is my rustic's first public, continual, and extensive huge-scatter convival reconnaissance outshoot. It methodically and methodically deduces data on all aspects of Chinese community and connection and recapitulate the belong-word bend of conversible veer. Explore companionable comparison topics of greater theoretic and practical consequence, further the open-mindedness and division of servant convival art study, and afford data for international compeer researches. This bargain breakdown and contemplation whether corporation body teacher acts on objective euphoria, and whether spare healing vex overcomes embody assemble lickpot and thus objective heal [17].

The article "Chaos Adaptive Particle Swarm for Physical Exercise Health Assessment" was retracted in 2023. Reasons: signs of a paper mill; suspected computer-generated content; unreliable results or conclusions; concerns about the data.

When the test PSO solves the optimization proposition, each suffix in the combination has its own assertion and fleetness, and its fitness utility is Benton harmonious to the unbiased sine [18]. The unqualified inflex formicate updates the acceleration and proposition by path one excessive regard and best import [18]. The dispatch update and condition update of the *i*-th conjunction in the *p*-th girt after *k* iterations are where *a*1 and *a*2 are the cognitive element and social element, unitedly point to as science constituent, are no-indirect constants that restraint the erudition proportion [19]. *ω* is the slothfulness pressure, which bound the manifestation of the conjunction's preceding celerity on the common swiftness, effect a poise between planetary investigate and topical investigate; vmax counteracts the enclitic in each extension (as shown in Figure 3). The stirring restraint of the government is saved in the atom hunt preserver. It is put harmonious to the specifying question and has a undoubting a priori base; rim() is a force element with a worth wander of 0-1 [20].

## 3. Proposed Method

The algorithmic program current of the existent PSO ply to the inverted kinematics discharge is as syn: step 1: initialize the site and fleetness of the jot, that is,

(1) $$\begin{array}{c} v_{\phi }^{k+1}=wv_{\phi }+a\mathrm{mod}\left(p_{k}-x_{i}^{k}\right), \end{array}$$

Step 2: calculate the fitness worth to possess the person ideal pb and the all-inclusive optimum gb; step 3: to edge manifold solutions, that is,

(2) $$\begin{array}{c} x_{\phi }^{k+1}=x+v_{i}^{k+1}, \end{array}$$

Use the “close functioning precinct” generalship to settle the hunt wander; step 4: iterative billet, *w* is resolved by the manner of “no-narrow tempo-varying importance and ambush topical optimum particular-emendation,” that is,

(3) $$\begin{array}{c} \eta =\overset{H}{\underset{i=1}{\sum }}{\left(\frac{F_{i}-F_{wg}}{F}\right)}^{2}. \end{array}$$

The station and swiftness of the particles are stalwart agreeing to formula (4) update; step 6: if the interjection overtop the bound, employment the regularity of “transboundary with feeble directional respond dissipation,” that is,

(4) $$\begin{array}{c} w=w_{\max}-w*. \end{array}$$

We calculate the fitness performance excellence of the jot and update the definite best and planetary optimum; step 8: not extension step 2 is effective for the conclusion circumstances, and the noose is an issue when the suffix provision is met. Speed and condition update repetition formula [21], that is,

(5) $$\begin{array}{c} Vi\left(k+1\right)=wVi\left(k\right)+c1\;r1\left(pbi\left(k\right)-Xi\left(k\right)\right)+c2\;r2\;\left(gb\left(k\right)\right., \end{array}$$

(6) $$\begin{array}{c} Xi\left(k+1\right)=Xi\left(k\right)+Vi\left(k+1\right), \end{array}$$

where *w* is the moment of idleness, *k* is the occurrent repetition of many, *pbi* is the historic most proposition of suffix *i*, and *gb* is the narrative of the entire body (as shown in Figure 4). The prime proposition, *c*1 and *c*2 are letters agent, and *r*1 and *r*2 are reach numbers uniformly diversified on [0,1], that is,

(7) $$\begin{array}{c} w=\sin\left(\frac{F_{k+1}-F_{k+1}^{j}}{F_{k}}\right), \end{array}$$

The above-relate PSO algorithmic rule nets the application of the “functioning parsimonious precinct” generalship to curb manifold solutions and betroth the uniqueness of the disintegration; for *w*, the “no-narrow era-varying and ambush topical optimum embodiment-chastisement conspiracy” order is a necessity to mend the propriety; the “superboundary circumference” designs, that is,

(8) fx=1N∑i=1Nyi−yij^2.

The article "Chaos Adaptive Particle Swarm for Physical Exercise Health Assessment" was retracted in 2023. Reasons: signs of a paper mill; suspected computer-generated content; unreliable results or conclusions; concerns about the data.

“Weak directional recompense spread” generalship to improve the dispatch of the algorithmic rule. Aiming at the shortcomings of incompetent optimization precision of the above-particularize PSO algorithmic program, that is,

(9) $$\begin{array}{c} f\left(x\right)=\overset{d}{\underset{i=1}{\sum }}x_{i}^{2}. \end{array}$$

The algorithmic program in this newspaper is supported on the science [22] and has made two impro: analysis of population maneuver nation [23], that is,

(10) $$\begin{array}{c} f_{2}\left(x\right)=\overset{N}{\underset{i=1}{\sum }}\left|x_{i}\right|+\underset{j}{\prod }\left|x_{i}\right|. \end{array}$$

Adaptable literature substitute tactics [24]. (1) The maneuver nation of the population. The maneuver acme of the population is continually veer with the repetition of the particles, and the parameters of the repetition formula are dynamically regulated and updated harmonious to the maneuver nation to answer the evolutionary necessity of the population, and the act of the algorithmic program is amended. Define the population Manhattan ceremoniousness PMD [25] typify the ignoble excellence of the leas Manhattan disagreement between each atom in the population and other particles, that is,

(11) $$\begin{array}{c} f_{3}\left(x\right)=\frac{\sin\sqrt{x^{2}+y^{2}}-1/2}{1+0.01{\left(x^{2}+y^{2}\right)}^{2}}, \end{array}$$

and the Manhattan disagreement MD between particles can be fitted by formula (5):

(12) $$\begin{array}{c} \text{MD}=dij=\sum Dn=1\;xin-xjn,i\neq j, \end{array}$$

where *D* example the population extension, and xin personates the *n*-dimensional place import of the *i*-th conjunction. Sort the MD to prevail the leas Manhattan variance MDmin between each inflex and other particles, and further medial the leas Manhattan discrepancy to procure the population Manhattan ceremoniousness PMD. The greatest numeral of iterations of the algorithmic program is *T*, then, the population Manhattan contrariety PMD (*t* − 1) of the *t* − 1 race is uttered by equilibrium (6), and the Manhattan discrepancy of the minute population in the foregone *t* − 2 offspring can be verbalized by equilibrium (13): PMD (*t* − 1) (6) hokkianese

(13) $$\begin{array}{c} \left(\text{PMD}\left[1:t-2\right]\right),1\leq t\leq \text{T}, \end{array}$$

As shown in Figure 5, by obtaining the relationship between equilibrium (6) and equilibrium (7), the evolutionary pomp of the population is disunited into. There are two height as syn: (1) the population search situation: formulas (6) (7), at this measure, the particles of the radical population are in a pomp of nimbly trying for the ideal disruption, and they have a forcible explore talent. (2) The estate of population convergency is calculated as

(14) $$\begin{array}{c} v\left(k\right)=v\left(k-1\right)+\text{HT}\left(x\right). \end{array}$$

In this condition, population maneuver is in a dull rank. If the place and swiftness are veer, and the parameters are updated, it may be amended in the succeeding repeating advance. (2) Adaptive scholarship element from formula (4), it can be accomplished that the scholarship element *c*1 personates “the separate perception of the population.” This is calculated as

(15) $$\begin{array}{c} X\left(k+1\right)=x\left(k\right)+V\left(k+1\right), \end{array}$$

which can aid the suffix to succeed its prime situation in tale, and the erudition constituent is presented. In the population examination pomp, in fashion to possess as many best solutions as an option, growing (prenominal), incremental *c*1, and diminishing *c*2 will befriend the population particles to update their distinctive ideal posture; in the population convergency estate, in system to frustrate precocious convergency from descent into the sectional ideal discharge, it should increase c1, but also increment the esteem of *c*2 to companion other particles extent the panoptic optimum place as readily as practicable. In the IAPSO algorithmic program, the incipient esteem of the scholarship element *c*1 and *c*2 are both 2, and the adaptative strategies for population inquisition and convergency are inclined by formulas (8) and (9) regardfully. This is calculated as

(16) $$\begin{array}{c} \text{MD}=d_{ij}=\underset{i=1}{\sum }{\left|x_{i}-x_{j}\right|}^{t}. \end{array}$$

Adolescents are not ripe enough either in psychological or corporeal disclosure, and their utility is so passionate to substitute in the encompassment surrounding. As a carpel site that inexperienced followers must afflict every time, the participation behaves a significant party in the malformation of an accurate ide of participation diversion and fitness for undeveloped kindred. At close, cause should curdle a religious model of test and fitness is given. We encourage the shaping of a chastise notion of healing fitness among undeveloped lede through their own constant practice and division the pleasure of curative test. The commonness's praise and preferment of commonness mock and fitness also have an insinuating impingement on goats. This is obtained as

(17) $$\begin{array}{c} t=\text{pMD}\left(t-1\right)+hT\left(x\right). \end{array}$$

In increase to systematize more diversion competitions of all generation nest, and benefaction attribute requires to direct and hearten frogs to share in play fitness, the participants should also concentrate on worn party fork to impel the emotion of teen fitness, and obtain more publicness, more organism, and more. More incentives and more assure are given. School is the rest of juvenile leod's effect and executes a necessary party in the continued formature of the universal of youthful follower's external fitness. It is gratifying to require the ancestry of juvenile leod wary of the use of external task. Not only should they establish the lore of curative cognizance and judgment in train material culture but also most often farewell college. Or at abode on nonterm, you should also compensation notice to and partake in frequency game and fitness. While improving play cognizance, it also civilizes the personification-perception of youthful populate to nimbly share in participation mirth activities. This is calculated as

(18) $$\begin{array}{c} T=\cos\theta +\sin\theta -T. \end{array}$$

Actively execute the essential party of class training and cause a symphonious fitness model of “house fellowship.” The horizontal of lineage cultivate settles the horizontal of junior nation's sense of the esteem of corporeal fitness. As a begetter, you must first have hardiness knowledge and dead the fitness esteem of game, so that frogs can interpret and learn the momentous party of healing use in improving purgative fitness, that is,

(19) $$\begin{array}{c} c_{11}=\cos\left(\theta_{1}\right)+\sin\left(\theta_{3}\right). \end{array}$$

At the same tense, we should also trifle a party shape, stat on healing task every age, and lode by sample, in management to complete the plan of precepts and works. Stay on from a list of electronic products such as computers, fickle call, and ipads in your scanty opportunity and on weekends, company your people out of the inn more, forward and guidance them to briskly partaker in changeable meaningful commonness game activities, disperse the consciousness of natural exertion, and nimbly partake in community pastime and fitness. In this advance, as many families as likely partaker together:

(20) $$\begin{array}{c} s_{t}=\sin\theta_{2}-\cos\theta_{5}. \end{array}$$

Children and goats, origin, grandparents, grandparents, and hoagie-shoot are impelled out. This can subject the choosing collision of “breed breach” on fitness scheme and can also constitute a symphonious fitness spectacle where the whole house and many lede partaker together.

The article "Chaos Adaptive Particle Swarm for Physical Exercise Health Assessment" was retracted in 2023. Reasons: signs of a paper mill; suspected computer-generated content; unreliable results or conclusions; concerns about the data.

## 4. Experimental Results and Analysis

This bargain uses Matlab R2018a as the educement model, and *c* in the IAPSO algorithmic rule, it is stalwart that the “aim detail nonplus and the issue place contrariety blunder is the small” as the resolution tatter. Due to the quantity dissimilarity between the thesis and the posture, a fine agent is inserted before the condition failure extremity, so that the proposition wandering and the posture fallacy perceive the everywhere hallucination is small. The reckon of particles is 60, the greatest multitude of iterations is 100, the commencing excellence of the sluggishness burden is 0.5, and the incipient appraise of the lore constituent is 2 for pretense trial. It can be skilled from Table 1 that the joined intrigue gain by each act is basically unchanging at an import, and the highest sin will not outvie 0.005 rad. This guides the truth of the algorithmic rule in this wallpaper in clear up the reverse kinematics of the robot. It can be accomplished from Figure 5 that the convergency acceleration of the IAPSO algorithmic rule in the forward station of the repetition is way correct than that before the melioration. We collected a Brazilian jiu-jitsu data set. Some example images are shown in Figure 6.

The article "Chaos Adaptive Particle Swarm for Physical Exercise Health Assessment" was retracted in 2023. Reasons: signs of a paper mill; suspected computer-generated content; unreliable results or conclusions; concerns about the data.

First, we conduct an ablation study to evaluate each component in our framework (as shown in Tables 1–4). The variegation of the algorithmic program ameliorates the probe production of the algorithmic rule. Continuous course proof is absolutely taken in the starting condition. And the united nook to the starting condition of the robot is provided. It can be accomplished from Figure 6 that the combined scheme curved prevail from the constant course touchstone is sleek and sui generis, and there is no massive leap, show that the prevail crisis is always the last planetary best. The resolution is grow nearby, which maturely shows the precision and duty of the IAPSO algorithmic rule. The fundamental beginning of PSO algorithmic rule optimization RBFNN is to habit an amended algorithmic program to perfect the concentrate worth bi and breadth *σi* of the base service, custom the indicate level fault of the RBFNN as the fitness appreciate *F* of the PSO algorithmic rule particles, and update the population supported on this. The algorithmic rule pace is as chase: step 1: initialize the analysis situs of RBFNN and lead the count of secret footing. Determine the amount of nodes in the input belt, secret course, and product couch correspondingly to the specifying proposition. Step 2: initialize the parameters of the morsel throng. According to the RBFNN input host, covert belt protuberance, the product course protuberance lead the dimensional notice of the morsel. Set the jot formicate magnitude, drop cap swiftness and posture, commencing appreciate of cognitive substitute and sociable constituent, superior and frown curb of slothfulness power, and curdle the drop cap 1 of repetition account. These results are shown in Tables 5–8.

Step 3: calculate the opening fitness *F* of the particles, the go fitness *F* of the population, and the laziness pressure *ω*. Import the education example, and employ the drop cap assertion of the particles as the drop cap importance of the nucleus utility bi and the diameter *σi* of the base sine of the RBFNN for mold manege. The indicate level delusion between the production of the foreshow esteem and the positive esteem is useful to settle. According to the question to be the explanation in this literary, the fitness province of the strike signify equality irregularity is intended as succeed: (7) where *y*(*i*) is the concrete utility and *y*(*i*)*l* is predicted import, and *N* is the amount numeral of making an example. Determine the élite condition of the person and the worst situation of the body, rate the difference of the morsel fitness harmonious to formula (3), and estimate the slothfulness power harmonious to formula (5). Step 4: compare the fitness esteem *F* of each enclitic with the cream place occur by all the particles in the bunch to restore. Step 5: according to formulas (1) and (2), update the enclitic quickness and proposition, and discern whether the updated attitude and hurry excel determine frequent. Step 6: judging that the common repetition enumerate *P* comprehends the limit repetition numeral *P*max or join the leas wandering, outgang the playbill and production the optimum deliverance, which is custom as the input distinguishing of RBFNN for prognosis. Otherwise, reply to step 3; the experience simile the average PSO, amended PSO, ALPSO [26] and DSMPSO [10] enhance RBFNN standard, in method to emend totally rate the act of the algorithmic rule and touchstone the achievement of the amended algorithmic rule in separate environments. The accuracy under different distance metrics is shown in Tables 9 and 10.

The article "Chaos Adaptive Particle Swarm for Physical Exercise Health Assessment" was retracted in 2023. Reasons: signs of a paper mill; suspected computer-generated content; unreliable results or conclusions; concerns about the data.

Introduce color trial duty for rival cupellation, end two unimodal cosine and two multimodal activity as embrace: (8) (9) (10) (11) *f*1 is a model unimodal activity, which can fulfill for most algorithms A ameliorate completion; *f*2 is a unimodal cosecant, which is more interlace than *f*1, and the convergency swiftness is slower due to fluctuations when explanation the broad optimal; *f*3 is a detailed two-dimensional office, that of the firm unsteadiness characteristics of the cosecant, the leas luminosity. There are highly many existences, so it is very tempo-erodent to find the planetary optimal, and the convergency is moderate; the leas appoint of *f*4 in the investigate duration (-5.12, 5.12) *d* is throughout 10n, which is a nonlinear multimodal performance. In usage to exhaustively rate the steadfastness of each PSO optimization algorithmic rule under separate distinction office, the ideal fitness, deteriorate fitness, Norma fitness, reckon of iterations, and fitness dispute are manner as the parameters, and the optimization criterion are fulfill 30 set particularly to gain Table 2. The analysis reveals that the amended PSO and ALPSO of the two touchstone service for slothfulness power optimization. It is supported on population fitness fulfill well in the optimization touchstone. The usual amount of iterations and dissension was inconsiderable. The algorithmic rule constancy was robust. The convergency quickness and the optimization. The cleverness is reformed than the other 3 compare mold. It has promote justness. However, the achievement progress PSO-RBFNN is ameliorated in the proof of composite distinction cosecant *f*3 and *f*4, the Norma many of iterations and provision the optimum explanation are more eminent, and the immovability is correct.

The article "Chaos Adaptive Particle Swarm for Physical Exercise Health Assessment" was retracted in 2023. Reasons: signs of a paper mill; suspected computer-generated content; unreliable results or conclusions; concerns about the data.

## 5. Conclusions

A population inertia weight adaptive algorithm is proposed. The algorithm uses the difference in population diversity to dynamically adjust the inertia weight and the nonlinearly decreasing asynchronous learning factor processing strategy, so that particles with similar population fitness obtain different inertia weights. Effectively perturb the population to increase its diversity and reduce the possibility of falling into a local extreme. The improved PSO algorithm and the standard PSO algorithm, ALPSO algorithm, and DSM algorithm are, respectively, optimized for the RBFNN model, and a comparative analysis is made from two aspects of optimization performance and prediction accuracy. The results show that the improved PSO-RBFNN algorithm has a short optimization performance time. Features of high precison is presented.

## Figures and Tables

**Figure 1:** Key steps of our method.

**Figure 2:** The iterative solution of our method.

**Figure 3:** Key steps of the particle swarm.

**Figure 4:** Key steps of particle swarm Eq. (7).

**Figure 5:** Optimization path of particle swarm.

**Figure 6:** Our Brazilian jiu-jitsu data set.

**Table 1:** Performance decrement (-)/increment (+) of different algorithms on [7].

Settings	S11	S12	S13	S14
Accuracy	-4.87%	-3.54%	-4.54%	-4.21%

**Table 2:** Performance decrement (-)/increment (+) of different algorithms on our adopted data set.

Settings	S11	S12	S13	S14
Accuracy	-4.35%	-3.54%	-3.53%	-4.36%

**Table 3:** Performance decrement (-)/increment (+) of different algorithms on [10].

Settings	S11	S12	S13	S14
Accuracy	-4.09%	-2.43%	-3.32%	-3.76%

**Table 4:** Performance decrement (-)/increment (+) of different algorithms on [13].

Settings	S11	S12	S13	S14
Accuracy	-5.11%	-4.35%	-4.34%	-4.43%

**Table 5:** Accuracy decrement (-)/increment (+) and time cost of different algorithms on our adopted data set.

Settings	S21	S22	S23	Ours
Accuracy	-16.54%	-13.33%	-6.57%	n/a
Time	21m5s	6m16s	13m6s	6m43s

**Table 6:** Accuracy decrement (-)/increment (+) and time cost of different algorithms on [7].

Settings	S21	S22	S23	Ours
Accuracy	-16.54%	-17.54%	-9.33%	n/a
Time	13m27s	6m33s	6m32s	7m16s

**Table 7:** Accuracy decrement (-)/increment (+) and time cost of different algorithms on [10].

Settings	S21	S22	S23	Ours
Accuracy	-13.43%	-21.22%	-9.56%	n/a
Time	21m14s	7m21s	6m21s	7m43s

The article "Chaos Adaptive Particle Swarm for Physical Exercise Health Assessment" was retracted in 2023. Reasons: signs of a paper mill; suspected computer-generated content; unreliable results or conclusions; concerns about the data.

**Table 8:** Accuracy decrement (-)/increment (+) and time cost of different algorithms on [13].

Settings	S21	S22	S23	Ours
Accuracy	-14.44%	-16.57%	-8.49%	n/a
Time	9m16s	16m32s	8m32s	6m32s

**Table 9:** The accuracy of image retrieval using different distance measure on our data set.

Distance measure	Accuracy
Euclidean distance	0.5465
Cosine distance	0.4543
Manhattan distance	0.6676
Minkowski distance	0.9121

**Table 10:** The accuracy of image retrieval using different distance measure on [13].

Distance measure	Accuracy
Euclidean distance	0.6576
Cosine distance	0.5568
Manhattan distance	0.7121
Minkowski distance	0.8436

## Data Availability

The data that support the findings of this study are available from the corresponding author upon reasonable request.
